# Efficacy and Safety Evaluation of Intramedullary Nail and Locking Compression Plate in the Treatment of Humeral Shaft Fractures: A Systematic Review and Meta-analysis

**DOI:** 10.1155/2022/5759233

**Published:** 2022-06-28

**Authors:** Yong Hu, Tianhui Wu, Baolin Li, Yongxiang Huang, Changqiang Huang, Yilin Luo

**Affiliations:** ^1^Departments of Orthopedics, Danzhou People's Hospital, Danzhou, 571700 Hainan, China; ^2^Departments of Orthopedics, People's Hospital of Wanning Hainan, Wanning, 571500 Hainan, China; ^3^Department of Trauma Surgery, Qionghai People's Hospital, Qionghai, 571400 Hainan, China

## Abstract

**Objective:**

The surgical treatment scheme of humeral shaft fracture is still controversial with no consensus reached. This meta-analysis was aimed at comparing the efficacy and safety of intramedullary nail (IMN) and locking compression plate (LCP) in the treatment of humeral shaft fractures.

**Methods:**

PubMed, Medline, Embase, Ovid, Cochrane Library, ISI Web of Science, Clinical Trials, and Chinese databases, including China National Knowledge Infrastructure Project, Wanfang database, and China biomedical abstracts database, were used to search the literature. Review Manager software was employed for statistical analysis and establishing forest and funnel maps. Categorical variables were measured by relative risk (RR), and standardized mean difference (SMD) was used to measure continuous variables. 95% confidence intervals were used for each variable. The modified Jadad scale, Newcastle-Ottawa scale, and Cochrane's bias risk tools were used to evaluate the bias and risk of eligible studies.

**Results:**

A total of 14 studies were included in the analysis with a total of 903 patients with humeral shaft fracture. Significant differences with regard to operation time (Std = −1.18, 95% CI: -2.14, -0.22, *Z* = 2.41, *P* = 0.02), blood loss (Std = −2.97, 95% CI: -4.32, -1.63, *Z* = 4.34, *P* < 0.001), and postoperative infection rate (RR = 0.32, 95% CI: -0.15, 0.68, *Z* = 2.98, *P* = 0.003) were noted between the IMN group and LCP group. In addition, the American Shoulder and Elbow Surgeon (ASES) score (Std = −0.22, 95% CI: -0.44, 0.01, *Z* = 2.08, *P* = 0.04) and the rate of shoulder and elbow function limitation (RR = 1.88, 95% CI: 1.06, 3.33, *Z* = 2.17, *P* = 0.03) between the 2 groups were also statistically significant. There were no significant differences in the rate of radial nerve injury, nonunion, delayed healing, and secondary operation between the two groups.

**Conclusion:**

IMN is superior than the LCP in terms of the operation time, intraoperative bleeding, and postoperative infection, suggesting its superiority in the humeral shaft fracture fixation. However, IMN is inferior to LCP in ASES score and shoulder elbow function limitation rate, indicating poor early postoperative functional recovery. More studies are required to evaluate and analyze the clinical efficacy between IMN and LCP regarding long-term function after artificial graft removal.

## 1. Introduction

Humeral shaft fractures are common in adult fractures, accounting for about 3% of all adult fracture types [1]. Controversies still exist about whether surgical intervention is needed for humeral shaft fractures. Surgical treatment is generally recommended for fractures with large displacement angles, multiple fractures, comminuted fractures, and fractures complicated with vascular and nerve injury [2, 3]. However, the failure rate and complications of the traditional plate and screw incision and internal fixation are high [4]. With the continuous improvement of surgical techniques and internal fixation implants, intramedullary nails (IMN) and locking compression plates (LCP) are widely used in the internal fixation of humeral shaft fractures with studies showing favorable clinical efficacy in both [5].

Several studies have compared the clinical efficacy of LCP and IMN with inconsistent results [6–8]. In addition, previous studies were limited by small study sample, suboptimal study quality, and inclusion of remote studies. The postoperative functional recovery results of this study were evaluated by the American Shoulder and Elbow Surgeon (ASES) score [9]. This study systematically assessed and meta-analyzed the literature on the efficacy of IMN and LCP in the treatment of humeral shaft fractures published in recent 20 years to better evaluate and compare the efficacy of these two schemes and provide a theoretical basis for clinical decision-making.

## 2. Materials and Methods

### 2.1. Literature Retrieval Strategy

Three independent researchers selected the database for literature retrieval following the principle of Cochrane. A total of 8 databases, including PubMed, Medline, Embase, Ovid, Cochrane Library, ISI Web of Science, Clinical Trials and China National Knowledge Infrastructure Project, Wanfang database, and China biomedical abstracts database, were employed for literature retrieval. The search terms, including “humeral shaft”, “humeral diaphyseal”, “humeral diaphysis”, “intramedullary nail”, and “plate”, were used individually or in combination. Any differences were settled through consultation and discussion.

### 2.2. Literature Selection

The inclusion criteria were as follows: (1) randomized controlled experimental studies or case-control studies published in 2000 or later; (2) LCP or IMN were used to treat humeral shaft fractures; (3) modified Jadad scale score ≥ 4 for randomized controlled trials or the Newcastle Ottawa mean scale (NOS) score ≥ 7 for case-control studies; (4) age ≥ 18 years; (5) the clinical data of patients are complete; and (6) there are corresponding data in the literature to calculate RR and STD values.

The exclusion criteria were as follows: (1) the types of literature were review, systematic evaluation, meta-analysis, case report, or editorial; (2) inclusion of patients <18 years old; and (3) nonprimary humeral shaft fractures, such as pathological fractures and old fractures after bone nonunion.

### 2.3. Data Extraction

In this study, two researchers independently extracted and screened data meeting the inclusion criteria for basic information and data extraction. The extracted data and characteristics included the following: literature title, first author, publication year, intervention measures, number of cases, operation time, intraoperative blood loss, complications, and ASES score. Data were extracted based on a broad selection of primary and secondary clinical outcomes from the literature included in this article. The third researcher checked the information and proofread the data to ensure the accuracy of the collected data.

### 2.4. Quality Evaluation

The modified Jadad scale, NOS, and Cochrane's bias risk tools were used to evaluate the bias and risk of eligible studies, as previously reported [10]. Study quality was evaluated with the modified Jadad scale that provides a semiquantitative rating from low quality (1-3 points) to high quality (4-7 points) based on summative score of 4 items, namely, randomization (2 points), concealment (2 points), blinding method (2 points), and withdrawal and dropouts (1 point). Similarly, the NOS scoring system had a total of 9 points, including selection of subjects (4 points), the comparability (2 points), and the measurement of exposure factors (3 points). The risk bias map was generated using Cochrane's bias risk tool.

### 2.5. Statistical Analysis

Review Manager software (version 5.4 of the Nordic Cochrane Centre, Copenhagen, Denmark) was used for statistical analysis and generation of the forest map and funnel map. Categorical variables were measured by relative risk (RR), and standardized mean difference (SMD) was used to measure continuous variables. 95% confidence intervals were used for each variable. Meta-analysis was conducted on the data included in the literature. The studies with clinical heterogeneity, which was assessed with the chi-square test and inconsistency index statistic (*I*^2^), were divided into subgroups. The test standard was *I*^2^ < 50%, *P* > 0.05. The fixed-effect model was used when the heterogeneity was low (*I*^2^ < 50%, *P* > 0.05). Otherwise, the random effect model was adopted. When *I*^2^ was inconsistent with the *P* value, the *P* value was used as the standard for selecting the processing model. A *P* < 0.05 denoted statistical significance.

## 3. Results

### 3.1. Search Results and Literature Quality Evaluation

The process of literature search and screening is shown in Figure 1. This study retrieved 1523 literature on IMN and plate internal fixation of humeral shaft fractures from the database. After screening according to the inclusion and exclusion criteria, 14 literatures were included in the analysis with a total of 903 patients, including 437 patients treated with IMN and 466 with LCP. Study quality is summarized in Table 1, and the risk bias diagram and summary are presented in Figure 2. A total of 12 RCT and 2 controlled clinical trials (CCT) were included in this study.

### 3.2. Operation Time

A total of 5 literature reported the operation time, and there was significant heterogeneity among the literature (*P* < 0.001, *I*^2^ = 95%). Therefore, a random-effect model was used. The combined Std, 95% CI, and effect amount *Z* were -1.18, (-2.14--0.22), and 2.41 (*P* = 0.02), respectively. As shown in Figure 3(a), the operation time of the IMN group was significantly shorter than that of the LCP group. Considering the large heterogeneity, the literature was screened for the latest 10 years and analyzed again. There was still significant heterogeneity among the literature (*P* < 0.001, *I*^2^ = 87%); thus, the random-effect model was used. The combined Std value, 95% CI, and combined effect amount *Z* were -1.63, -2.33--0.93, and 4.55 (*P* < 0.001), respectively. The operation time in the IMN group was shorter than that in the LCP group in recent ten years (Figure 3(b)).

### 3.3. Intraoperative Blood Loss

Four studies reported intraoperative blood loss, and there was significant heterogeneity among the literature (*P* < 0.001, *I*^2^ = 96%). The combined Std value was -2.97, 95% CI was (-4.32, -1.63), and the combined effect amount *Z* was 4.34 (*P* < 0.001). The results showed that the intraoperative blood loss in the IMN group was less than that in the LCP group (Figure 4).

### 3.4. American Shoulder and Elbow Surgeon (ASES) Score

Seven studies reported the ASES score, and no significant heterogeneity was found among the literature (*P* = 0.61, *I*^2^ = 0%). The combined Std value was -0.22, 95% CI was (-0.44, 0.01), and the combined effect amount *Z* was 2.08 (*P* = 0.04). The ASES score of the IMN group was statistically lower than that of the LCP group (Figure 5(a)). Begg's test showed no publication bias, as shown in Figure 5(b).

### 3.5. Incidence of Nonunion

The incidence of bone nonunion was reported in 13 studies with no significant heterogeneity (*P* = 1.00, *I*^2^ = 0%). The combined RR value was 0.83, 95% CI was (0.47, 1.46), and the combined effect amount *Z* was 0.63 (*P* = 0.53). No significant difference in the incidence of bone nonunion between the two groups was noted (Figure 6(a)). Begg's test showed no publication bias (Figure 6(b)).

### 3.6. Incidence of Radial Nerve Injury

The fixed model was adopted since all the 13 studies that reported the incidence of radial nerve injury showed no significant heterogeneity (*P* = 1.00, *I*^2^ = 0%). The combined RR value was 0.90, 95% CI was (0.51, 1.57), and the combined effect amount *Z* = 0.38 (*P* = 0.70). There was no significant difference with regard to the incidence of radial nerve injury between the two groups, as shown in Figure 7(a). Begg's test showed no publication bias (Figure 7(b)).

### 3.7. Incidence of Postoperative Infection

No significant heterogeneity was found in the 12 literature (*P* = 0.96, *I*^2^ = 0%) that reported the incidence of postoperative infection. The combined RR, 95% CI, and effect amount *Z* was 0.32, 0.15-0.68, and 2.98 (*P* = 0.003), respectively. The postoperative infection rate of the IMN group was significantly lower than that of the LCP group (Figure 8(a)). Begg's test showed no publication bias (Figure 8(b)).

### 3.8. Incidence of Reoperations

No significant heterogeneity was found in the 11 literature (*P* = 0.41, *I*^2^ = 3%) that reported the incidence of reoperations. The combined RR value was 1.14, 95% CI was (0.58, 2.25), and the combined effect amount *Z* = 0.37 (*P* = 0.71).  Figure 9(a) shows no significant difference in the incidence of secondary surgery between the two groups. Begg's test showed no publication bias (Figure 9(b)).

### 3.9. Incidence of Delayed Healing

A total of 10 studies reported the incidence of delayed healing, and no significant heterogeneity was found (*P* = 0.68, *I*^2^ = 0%). The combined RR value was 1.39, 95% CI was (0.69, 2.80), and the combined effect amount *Z* = 0.91 (*P* = 0.36). No significant difference in the incidence of delayed healing was observed between the two groups, as shown in Figure 10(a). Begg's test shows no publication bias (Figure 10(a)).

### 3.10. Incidence of Shoulder/Elbow Joint Limitation

No significant heterogeneity was found in the 9 literature (*P* = 0.21, *I*^2^ = 30%) that reported the incidence of should/elbow joint limitation. The combined RR value was 1.88, 95% CI was (1.06, 3.33), and the combined effect amount *Z* = 2.17 (*P* = 0.03). The incidence of shoulder/elbow joint limitation in the IMN group was significantly higher than that in the LCP group (Figure 11(a)). Begg's test showed no publication bias (Figure 11(b))].

## 4. Discussion

Patients with humeral shaft fracture are often complicated by neurovascular injury, open fracture, combined elbow forearm fracture, and compound multiple injuries [22, 23]. There are still debates about the optimal management scheme for humeral shaft fracture in the clinic. At present, the main surgical methods include open reduction and internal fixation and intramedullary nail fixation. LCP is widely used in open reduction and internal fixation [5]. Some systematic evaluations and meta-analyses have compared the treatment of humeral shaft fractures with LCP and IMN with inconsistent findings [24–27]. Ozan et al. found that IMN was safer and more applicable and effective than steel plate in treating type A humeral shaft [28]. In a meta-analysis published in 2010 by Heineman et al., it was noted that there were no significant differences in the incidence of postoperative complications, bone nonunion, postoperative infection, radial nerve injury, and reoperations [29]. A plausible explanation for the inconsistencies is that the studies included in the meta-analysis are of mixed quality. Therefore, this study included only RCTs with a modified Jadad scale score ≥ 4 or CCT with a NOS ≥ 7.

The main comparative parameters of the two groups included the incidence of nonunion, iatrogenic radial nerve injury, and postoperative infections. According to relevant research reports, the incidence of bone nonunion was as high as 3-20% [30]. In a study of 325 surgically treated adult humeral shaft fractures, Claessen et al. [31] found that the surgical approach, especially the open approach, was significantly related to iatrogenic radial nerve injury. Ma et al. found no significant difference between IMN and LCP with regard to the success rate of fracture healing, incidence of radial nerve injury, and postoperative infection [24]. This study demonstrated that IMN reduced postoperative infection as compared with LCP, but there were no significant differences in bone nonunion and radial nerve injury. We also reported increased rate of postoperative infections in the LCP group than that in the IMN group, which may be attributed to the fact that the LCP approach is more traumatic with increased intraoperative blood loss and longer operation duration. The similar success rate of fracture healing and incidence of radial nerve injury also support the application of IMN. However, many controversies still exist about the postoperative infection rate and fracture healing rate between the two. For example, Heineman et al. suggested that applying steel plate to humeral shaft fracture is more likely to reduce the incidence of complications [32], whereas Ozan et al. reported that the incidence of bone nonunion in the IMN group was lower in only one patient [28]. Therefore, future high-quality clinical research should be carried out to strengthen reporting homogeneity during follow-up.

The parameters of efficacy evaluated included operation time, delayed fracture healing, reoperation rate, and intraoperative blood loss. The analysis of this study showed that IMN was superior to the LCP group in operation time and blood loss. Although the included studies have high heterogeneity in operation time and blood loss, which may be related to the significant fluctuation of clinicians' technical level, the analysis results still supported that IMN was advantageous in operation time and blood loss. Interestingly, when only studies published in the recent ten years were included, the operation time of the IMN group was significantly shorter than that of the LCP group, which is different from that reported previously by Wen et al. These discrepancies may be related to the application of IMN and rapid development of surgical techniques [27]. Although the difficulty of open internal reduction is reduced under direct vision, the preparation time is generally much longer. After the widely used intramedullary nail in the clinic, the technology is mature. Although IMN reduction is technically more challenging than LCP, skilled surgeons could still perform the operation with dramatically reduced time as compared with that of the ten years ago. IMN is also characterized by small incisions with reduced intraoperative blood loss. This study also found no significant difference in delayed fracture healing and reoperation rate, which was consistent with previous studies.

This study showed that the IMN group was inferior to LCP group in terms of ASES score and shoulder/elbow limitation rate. This is consistent with the results of the previous meta-analysis that have also shown that using steel plates reduces the probability of postoperative shoulder joint limitation. Meanwhile, it has been suggested that IMN was more likely to cause apparent shoulder joint dysfunction in elderly patients [33, 34]. However, these studies are limited by short follow-up time, and few studies have compared and analyzed the functional recovery of the latter after removing artificial grafts.

Our study strength was inclusion of high-quality studies. A total of 14 studies with 927 subjects were included in this paper, which was the most systematic and comprehensive analysis so far. In addition, the updated clinical research has also brought additional research and analysis conclusions from previous studies. The heterogeneity of some data was wide, suggesting that the clinical results are constantly adjusted with the progress of technology. In the future, it is still necessary to carry out multicenter prospective randomized controlled trials with large sample size to conclusively determine the efficacy and safety of IMN vs. LCP for treating humeral shaft fractures.

To sum up, although IMN is superior to LCP in the fixation of humeral shaft fracture, it is limited by suboptimal early postoperative functional recovery. In the future, additional studies are entailed to evaluate and analyze the clinical efficacy between IMN and LCP with regard to long-term function after artificial graft removal.

## Figures and Tables

**Figure 1:** Flow chart of literature screening.

**Figure 2:** Quality of research methodology and risk assessment of bias included in the literature.

**Figure 3:** Meta-analysis forest of operation time. (a) Meta-analysis forest of operation time in the IMN group and LCP group. (b) Meta-analysis forest of operation time in the IMN and LCP groups in recent ten years.

**Figure 4:** Meta-analysis of intraoperative blood loss in the IMN group and LCP group.

**Figure 5:** Meta-analysis of ASES scores in the IMN group and LCP group. (a) Forest figure. (b) Funnel figure.

**Figure 6:** Meta-analysis of the incidence of bone nonunion in the IMN group and LCP group. (a) Forest figure. (b) Funnel figure.

**Figure 7:** Meta-analysis of the incidence of radial nerve injury in the IMN group and LCP group. (a) Forest figure. (b) Funnel figure.

**Figure 8:** Meta-analysis of postoperative infection rate in the IMN group and LCP group. (a) Forest figure. (b) Funnel figure.

**Figure 9:** Meta-analysis of the incidence of secondary surgery in the IMN group and LCP group. (a) Forest figure. (b) Funnel figure.

**Figure 10:** Meta-analysis of delayed healing rate in the IMN group and LCP group. (a) Forest figure. (b) Funnel diagram.

**Figure 11:** Meta-analysis of the incidence of shoulder elbow joint limitation in IMN group and LCP group. (a) Forest figure. (b) Funnel figure.

**Table 1:** Basic characteristics and document quality scores of included documents.

Study	Study design	Study assessment scale	IMN amounts	LCP amounts	Total amounts
Akalın et al. [11]	RCT	6	30	33	63
Bisaccia et al. [8]	CCT	7	26	32	58
Zhao et al. [7]	CCT	8	59	63	122
Fan et al. [2]	RCT	4	30	30	60
Zhang et al. [12]	RCT	4	50	50	100
Wali et al. [13]	RCT	4	25	25	50
Wang et al. [14]	RCT	4	22	23	45
Chaudhary et al. [15]	RCT	6	50	50	100
Li et al. [16]	RCT	4	22	23	45
Singisetti et al. [17]	RCT	5	25	20	45
Putti et al. [18]	RCT	4	16	18	34
Changulani et al. [19]	RCT	5	23	24	47
Mccormack et al. [20]	RCT	4	21	23	44
Chapman et al. [21]	RCT	4	38	46	84

RCT: randomized controlled trial; CCT: controlled clinical trial; study assessment scale: RCT study uses the modified Jadad scale; CCT study uses Newcastle-Ottawa scale.

## Data Availability

The data used to support the findings of this study are included within the article.
